The article "Correlation Analysis of Serum Pepsinogen, Interleukin, and TNF-α with Hp Infection in Patients with Gastric Cancer: A Randomized Parallel Controlled Clinical Study" was retracted in 2023. Reasons: signs of a paper mill; compromised peer review; unreliable results or conclusions.

# Correlation Analysis of Serum Pepsinogen, Interleukin, and TNF-*α* with Hp Infection in Patients with Gastric Cancer: A Randomized Parallel Controlled Clinical Study

**DOI:** 10.1155/2022/9277847

**Published:** 2022-09-14

**Authors:** Shunxin Hao, Minyue Shou, Jing Ma, Yongqian Shu, Yuanyuan Yu

**Affiliations:** ^1^Department of General Surgery, Wuhan University of Science and Technology Hospital, China 430065; ^2^The First Affiliated Hospital of Nanjing Medical University (Department of Oncology), China 210029; ^3^Zhongshan Hospital Affiliated to Fudan University, China 200032; ^4^Department of Geriatrics, Wuhan Hospital of Traditional Chinese Medicine, 49 Lihuangpi Road, Jiangan District, Wuhan City, Hubei Province, China

## Abstract

**Background:**

Gastric cancer pathological biopsy and visual examination have been the gold standard for gastric cancer diagnosis, but their operation is costly, demanding, and risky, so it is especially important to find an effective examination method in clinical practice.

**Aims:**

To investigate the correlation between serum pepsinogen I (PGI), pepsinogen II (PGII), pepsinogen I and II ratio (PGR), IL-6, and TNF-*α* and Helicobacter pylori (Hp) infection in patients with gastric cancer.

**Materials and Methods:**

Fifty patients with Hp-infected gastric cancer admitted to the Department of Gastroenterology of our hospital from January 2019 to December 2021 were selected for the study as the observation group, and another 50 patients without Hp-infected gastric cancer were selected as the comparison group to compare the correlation analysis of PGI, PGII, PGR, IL-6, and TNF-*α* with Hp infection between the two groups after admission and treatment.

**Results:**

After measurement, PGI and PGII in the observation group were significantly lower than those in the comparison group, and TNF-*α*, IL-18, and IL-6 in the observation group were significantly higher than those in the comparison group, and the comparative differences were all statistically significant (*P* < 0.05). The results of multivariate logistic regression model analysis of independent risk factors for gastric cancer showed that IL-18, hs-CRP, and tumor necrosis factor- (TNF-) *α* were risk factors for Hp infection in gastric cancer.

**Conclusion:**

The expression of IL-18, hs-CRP, and TNF-*α* factors in Hp-infected gastric cancer patients is correlated. IL-6, IL-18, and TNF-*α* are involved in the entire process from the onset to the development of Hp-positive gastric mucosal inflammation in patients, which is of great value in the diagnosis of gastric cancer and helps to assess the degree of progression and prognosis of gastric cancer.

## 1. Introduction

Epidemiological surveys in recent years have shown that the global morbidity and mortality of gastric cancer have been decreasing year by year, but it is still a common clinical malignant tumor [1]. The incidence of gastric cancer in my country ranks first among various malignant tumors, and it also accounts for 35% of the global incidence [2]. Epidemiological surveys have shown that with age, the incidence of H. pylori infection will continue to increase [3]. In recent years, studies have confirmed that H. pylori is closely related to the occurrence of gastric cancer, because H. pylori can cause damage to the gastrointestinal mucosa and promote the regeneration of gastrointestinal cells, thereby increasing the risk of injury [4]. H. pylori infection can increase the generation of oxygen free radicals, which leads to the peroxidation of gastric mucosal epithelium, which induces symptoms such as acid reflux, nausea, upper abdominal pain, and belching and is closely related to the incidence of gastric cancer [5]. Interleukin-18 (IL-18), high-sensitivity C-reactive protein (hs-CRP), and tumor necrosis factor-*α* (TNF-*α*) are highly sensitive markers of inflammatory factors [6]. Studies have confirmed that these inflammatory factors can induce and aggravate inflammatory responses, and IL-18 is involved in the occurrence and development of various malignant tumors including gastric cancer through various mechanisms [7]. After the inflammatory reaction, due to the continuous increase of free radicals and the generation of superoxide, the cells undergo peroxidative damage, resulting in long-term cellular tumors and gastric cancer [8]. H. pylori is a Gram-negative bacterium with multiple genotypes and secretes a variety of exogenous toxins [9]. It can damage the gastric mucosal epithelium, and the damage mechanisms include cell DNA damage, mitochondrial base expression affecting gastric mucosal epithelial cells, and cell proliferation disorders .

Studies have shown that H. pylori is closely related to gastritis, peptic ulcer, and gastric cancer. H. pylori infection is an important factor in the incidence of gastric cancer and is listed as the first carcinogen by the World Health Organization [10]. The relationship between H. pylori infection and cell proliferation and apotheosis is a current research hotpot [11]. The stability of the gastric environment requires a balance between proliferation and apotheosis of gastric colossal cells. Although the rate of cell loss caused by apotheosis is comparable to the rate of new cell formation, H. pylori infection will affect this balance and lead to the occurrence of many gastric diseases [12]. It has been suggested that Hp infection affects PG changes, and Hp infection plays an important role in gastric carcinogenesis, but its exact mechanism of action is not clear. Hp is a trigger for a number of diseases, and Hp activates disease cells, causing them to accumulate in the gastric mucosal tissues, creating a mediated inflammatory response, and the levels of cytokines in chronic gastritis vary significantly. The higher the level of Hp in the patient, the more severe the degree of infection of the patient's gastric mucosa, and the degree of erosion of the Hp-positive gastric mucosa by disease cells has an important relationship with the density of Hp. Peptic ulcer is a common gastrointestinal disease with a complex etiology, and Hp infection is one of its important causes. We believe that Hp infection affects PG changes and Hp infection plays an important role in gastric carcinogenesis, but its specific mechanism of action is not clear. The reason why Hp affects PG changes and causes cancer may be related to chronic inflammatory stimulation of Hp leading to atrophic intestinalization of gastric tissues and damage to PG genes, and some scholars believe that it is related to the host's own immune disorder caused by Hp. In this study, 100 patients admitted to our hospital from January 2016 to January 10, 2020, were selected for exploration and analysis and the correlation analysis of serum pepsin, IL-6, and TNF-*α* with Hp infection in patients with gastric cancer. The report is as follows.

## 2. Material and Methods

### 2.1. Research Object

Fifty cases of Hp-infected gastric cancer patients admitted to the Department of Gastroenterology of our hospital were selected for the study as the observation group, and another 50 cases of patients without Hp infection were selected as the comparison group. Inclusion criteria [13]: (i) after gastroscopic biopsy histopathological examination, pathology and imaging consistent with the diagnosis of gastric cancer; (ii) age 18-65 years, no history of special medication (gastric mucosal protective agents, nonsteroidal anti-inflammatory drugs, acid suppressants, and antibacterial drugs) in the previous 2 months, all selected patients accepted and voluntarily joined the experiment; (iii) no history of relevant vaccinations, approved by the hospital ethics committee and those who signed the informed consent. Exclusion criteria: (i) with infectious diseases, (ii) with severe liver and kidney impairment, and (iii) with mental illness (interfering with our study or affecting the results of the trial).

### 2.2. Methods

Serum-related factor assay: 2 ml of fasting elbow venous blood was collected from both groups in the early morning, and the serum was separated after centralization at 3000 r/min for l0min, and the level of CRP was measured by enzyme-linked immunodeficient assay kit (Bioengineering Shanghai Co., Ltd.); IL-18 and TNF-*α* were measured by IMMU-NITE1000 luminescence analyzer (Thermo Fisher) (kit: Institute of Radiology and Immunology, PLA General Hospital). The 2000 luminescence instrument from Abbott and the accompanying PGI and PGII reagents were used to determine PGI and PGII levels and calculate the PGI/PGII (PGR) ratio, which was determined by the luminescence method; patients were kept in a fasting state before undergoing gastropod, 3 ml of venous blood was collected, serum was separated to obtain serum and tested, and the degree of gastric colossal inflammation was measured. The degree of inflammation of the gastric mucous was observed with a low-mounted microscope, and the values of IL-6, IL-18, and TNF-*α* were recorded and analyzed.

Hp assay: the anti-Hp antibody characterization kit (Shanghai Changchun Technology Co., Ltd., enzyme-linked immunodeficient assay) was used to detect the level of Hp-IgG antibody in the serum of the two groups of patients.

### 2.3. Statistical Analysis

All statistical data in this study were entered into Excel software by the first author and the corresponding author, respectively, and the statistical processing software was SPSS 25.0 for calculation. Repeated measures analysis of variance between groups was used to measure the measurement expressed as mean ± standard deviation (*X* ± *S*). Count data expressed as a percentage (%) were tested by *χ*^2^. Univariate and logistic multivariate regression analysis was used to compare the influencing factors, and the risk factors with significant differences were screened. Correlation test used logistic regression linear correlation analysis. Included data that did not conform to a normal distribution were described by *M* (QR), using the Mann–Whitney test. All statistical tests were two-sided probability tests. The statistical significance was *P* < 0.05.

## 3. Results

### 3.1. Comparison of Baseline Data

The differences in mean age, gender, lesion diameter, tumor classification, and body mass index between the two groups were not statistically significant (*P* > 0.05). See Table 1.

### 3.2. Serum Index Comparison

After measuring, PGI (95.76 ± 3.14) and PGII (16.36 ± 4.90) in the observation group were significantly lower than those in the comparison group, and TNF-*α* (82.28 ± 4.24), IL-18 (19.76 ± 3.14), and IL-6 (9.13 ± 1.01) in the observation group were significantly higher than those in the comparison group, and the differences were statistically significant (*P* < 0.05). See Figure 1.

### 3.3. Comparison of Gastric Cancer Stage and Related Indicators

The higher clinical stage of gastric cancer led to higher serum gastrin-17, CEA, and CA199 levels and lower pepsinogen I levels, and the comparative differences were statistically significant (*P* < 0.05). However, the differences of pepsinogen I/pepsinogen II and H. pylori positivity rates in patients with different gastric cancer stages were not statistically significant (*P* > 0.05). See Figure 2.

### 3.4. Multiword Regression Analysis

The variables with significant differences were assigned, namely, IL-18, CA199, CEA, hs-CRP, and TNF-*α* (normal = 1, abnormal = 0). The results of multivariate logistic regression model analysis of independent risk factors for gastric cancer showed that IL-18, hs-CRP, and TNF-*α* were risk factors for Hp infection in gastric cancer, and the comparative differences were all statistically significant (*P* < 0.05). See Table 2.

## 4. Discussion

Hp infection is an important trigger of chronic gastritis and peptic ulcer, and research data show that some immune mechanisms and inflammatory responses play an important role in the pathogenesis of gastric mucosa, and nowadays, diseases due to cytokine triggers are getting more and more attention [14]. Hp-positive chronic gastritis and peptic ulcer make some cells in patients to form an immune response, in which endocrine secretion of serum IL-6, IL-8, and TNF-*α* and other cytokines is endocrine raised [15]. Hp is the trigger of some diseases, Hp activates disease cells and causes them to accumulate in the gastric mucosal tissue, forming a mediated inflammatory response, and the levels of cytokines in chronic gastritis differ significantly [16]. The higher the level of Hp in the patient, the more severe the degree of infection of the patient's gastric mucosa, and the degree of erosion of the Hp-positive gastric mucosa by the disease cells has an important relationship with the density of Hp [17]. Peptic ulcer is a common gastrointestinal disease with a complex etiology, and Hp infection is one of its important causes [18].

We found that Hp can secrete a large number of pathogenic factors via regulation of relevant signaling pathways, and long-term persistent Hp infection induces immune and inflammatory responses and produces carcinogenic substances, thus playing a role in the progression of precancerous diseases [19]. In addition, persistent Hp infection leads to an increased rate of DNA damage, and inflammation can lead to the production of large amounts of superoxide and free radicals, reducing the concentration of vitamin C in the gastric juice [20]. This makes the cells less tolerant to oxidative damage and prone to peroxidative damage [21]. The possible mechanisms linking Hp infection to the development of gastric cancer are considered to include the following: oxidative damage, type of Hp strain, genetic variants and differences in their expression, and abnormal kinetics related to gastric mucosal epithelial cells [22–25].

Our study showed showing that serum IL-6 and 1L-18 has an important factor in gastrointestinal diseases and also provides a diagnostic basis for patients with early gastric cancer [26]. Elevated serum IL-6 levels have been reported to be positively correlated with the development of bone tumors, and higher levels of IL-6 have been found in tumor cells and tumor-associated macrophages, and it has been found that tumor cells may produce higher levels of IL-6 during proliferation, invasion, or metastasis [27]. Elevated serum IL-6 levels were positively correlated with tumor load and disease progression, and IL-6 levels were significantly elevated in patients with gastric cancer with lymph node metastasis [28]. Serum pepsinogen, an endoproteinase with digestive function, is divided into two subgroups, PGI and PGII, according to immunology and biochemistry [29]. Among them, PGI is mainly expressed in cervical mucus cells and principal cells of the gastric fundus and is especially highly expressed in the gastric mucosa of embryos [30]. Among them, PGII is mainly expressed with all duodenal Brunner's gland and gastric glands and to a lesser extent in prostate and pancreas [31]. Most of the synthesized pepsinogen is secreted into the gastric lumen and activated into pepsin by the action of acidic gastric juice, and the pepsinogen that enters the circulation is very stable [32]. The measurement of serum pepsinogen changes can reflect the degree of gastric mucosal lesions and differentiation, which is beneficial for the early diagnosis of gastric cancer and is important for the prevention of gastric cancer, and it is also considered to be the best serological indicator for the histology of gastric mucosa [33]. Therefore, it is considered that serum pepsinogen can be used for the initial screening of gastric cancer and as an ideal tumor marker for the diagnosis of gastric cancer [34].

In our study, pepsinogen I and pepsinogen II in the observation group were significantly lower than those in the comparison group, and TNF-*α* and IL-6 in the observation group were significantly higher than those in the comparison group after measurement. The findings may suggest that elevated IL-6 levels may be an indicator of further deterioration of gastric cancer patients or suggest that the tumor may metastasize, suggesting appropriate therapeutic measures to control the development of the disease, and the experimental results have some clinical guidance [35]. TNF-*α* is one of the cytokines with the strongest antitumor effect, and both in vivo and ex vivo experiments have shown that TNF-*α* has very significant antitumor effect. Patients with higher tumor TNF-*α* values are more prone to metastasis and recurrence after treatment [36]. Therefore, TNF-*α* can be used as an important marker for tumor recurrence and metastasis, as well as an indicator for identifying pretumor lesions, and the experimental results are consistent with the literature [37]. The mean value of serum TNF-*α* in patients with lymph node metastasis from gastric cancer was nearly 6-fold higher than normal, and the mean value of serum TNF-*α* in patients with postoperative recurrence was nearly 3-fold higher than normal, which may be due to increased tumor load and excessive release of TNF-*α* from activated lymphocytes in vivo, resulting in increased serum TNF-*α* levels [38].

Our study also suggests that the determination of TNF-*α* activity in serum of gastric cancer patients, like the determination of IL-6, can be used as an adjunct to observe the progress of patients' disease and judge the deterioration or tumor metastasis, which has some reference value for clinicians [39]. Since the level of serum pepsinogen directly reflects the function of gastric mucosa, the significant decrease in serum pepsinogen I level in gastric cancer patients suggests that the secretion capacity of gastric mucosa of gastric cancer patients is reduced, and the significant decrease in serum pepsinogen I level in gastric cancer patients is related to atrophy, intestinalization, and reduced secretion of gastric mucosa in gastric cancer patients [41]. There was no statistically significant change in serum PC II levels in gastric cancer patients, which may be related to the wide distribution of 11 cells secreting pepsinogen [42]. A significant decrease in serum pepsinogen I is clinically important for the monitoring of early gastric cancer, and pepsinogen I and pepsinogen II are elevated in patients with gastric ulcer, whereas serum PGI and pepsinogen II are significantly lower in patients with cancer [43].

Multifactorial logistic regression analysis in our study showed that serum pepsinogen I, TNF-*α*, and IL-6 in gastric cancer were independent risk factors for Hp infection as a complication of gastric cancer. It indicates that serum pepsinogen and IL-6 tests can predict Hp infection in gastric cancer [44]. We believe that serum pepsinogen and IL-6 predicting Hp infection in gastric cancer also has some limitations to some extent, but the combination of separate tests can be used to improve the sensitivity of detection, early detection of Hp infection in gastric cancer, early intervention, and improve the survival rate of patients [45]. Existing clinical studies have shown that peripheral blood of gastric cancer patients showed a significant increase in serum pepsinogen, IL-6, which was correlated with tumor diameter and highly pelvic lymph node metastasis in gastric cancer patients, which is considered a factor associated with gastric cancer development and prognosis. IL-6 is a functional protein, mainly expressed by macrophages and epidermal cells, and is a common inflammatory factor with immunomodulatory and inflammation-mediated response. It has an important role in tissue injury and repair stages. Studies have shown phantom that the expression capacity of IL-6 is significantly lower in healthy humans than in patients with gastrointestinal diseases. IL-8 is mainly secreted by macrophages and epidermal cells and is also a common inflammatory factor with inflammation-mediating and endothelial cell proliferation effects, accelerating angiogenesis role. IL-8 has an important role at the beginning of the pathogenesis of diseases such as insulin, inflammation, and xanthogranuloma. TNF-*α* is a class of cytokines with multiple activities, which can overactivate leukocytes. This increases the adhesion of leukocytes to endothelial cells and makes leukocytes more easily phagocytized. The current study showed that when patients were infected with Hp, the concentration of TNF-*α* in the organism was significantly increased.

In conclusion, the expression of IL-18, hs-CRP, and TNF-*α* factors in Hp-infected gastric cancer patients is correlated, and IL-6, IL-18, and TNF-*α* are involved in the entire process from the onset to the development of inflammation in the Hp-positive gastric mucosa of patients, which is of great value in the diagnosis of gastric cancer and helps to assess the degree of progression and prognosis.

## Figures and Tables

**Figure 1:** Comparison of serum indicators. In this study, the statistics of the pain VAS scores of the two groups of patients were entered into Excel software by the first and corresponding author, respectively, and the included data were tested using the Shapiro-Wilk method of mean ± standard deviation of the measured data conforming to a normal distribution. And independent sample or paired sample *t*-tests were implemented between or within groups. PGI and PGII in the observation group were significantly lower than those in the comparison group, and TNF-*α*, IL-18, and IL-6 in the observation group were significantly higher than those in the comparison group, and the comparative differences were all statistically significant (*P* < 0.05).

**Figure 2:** Comparison of gastric cancer staging and related indicators. In this study, statistics of pain VAS scores for both groups were entered into Excel software by the first and corresponding authors, respectively, and measures of gastrin-17, CEA, CA199, PGI, and PGI/PGII were tested for inclusion by the Shapiro-Wilk method of mean ± standard deviation. And independent sample or paired sample *t*-tests were implemented between or within groups, and HP-positive rate count data were expressed as whole numbers and found by chi-square test. Higher clinical stage of gastric cancer resulted in higher serum gastrin-17, CEA, and CA199 levels and lower PGI levels, all with statistically significant differences in comparison (*P* < 0.05). However, the differences in PGI/PGII and HP-positive rates were not statistically significant in patients with different gastric cancer stages (*P* > 0.05).

**Table 1:** Comparison of baseline information between the two groups of patients.

Group	Average age (years)	Gender (male/female)	Lesion diameter (cm)	Body mass index (kg/m^2^)	Tumor classification	
					Gastric body cancer	Gastric sinus cancer
Comparison group (50)	69.83 ± 5.13	23/27	4.50 ± 1.25	22.32 ± 1.16	22	28
Observation group (50)	68.72 ± 3.16	26/24	4.40 ± 1.01	22.11 ± 1.10	21	29
*t*	1.303	0.360	0.440	0.929	0.041	
*P*	0.196	0.548	0.661	0.355	0.840	

**Table 2:** Multiword logistic regression analysis.

	*b*	SE (*b*)	Wald	*P*	OR	OR 95% CI
IL-18	2.026	0.952	4.370	0.023	7.656	1.110-5.760
CA199	-0.203	0.708	0.053	0.742	0.761	0.150-3.780
CEA	0.502	0.710	0.376	0.527	1.633	0.330-7.970
hs-CRP	4.932	1.409	10.412	0.003	1.910	7.021-217.402
TNF-*α*	-1.915	0.908	4.309	0.023	0.110	0.020-0.840

## Data Availability

No data were used to support this study.
